The article "Antineoplastic Effects of Ankaferd Hemostat" was published in 2022. Journal: Biomed Res Int.

# Antineoplastic Effects of Ankaferd Hemostat

**DOI:** 10.1155/2022/2665903

**Published:** 2022-08-02

**Authors:** Umit Yavuz Malkan, Ibrahim Celalettin Haznedaroglu

**Affiliations:** Hacettepe University, Faculty of Medicine, Department of Hematology, Ankara, Turkey

## Abstract

**Materials and Methods:**

Up to June 2022, literature searches were performed using the internet search engines Medline, Google Scholar, and Embase: Ankaferd. PRISMA flow diagram described the Ankaferd search.

**Results:**

ABS have important effects in several cellular processes, like control of the cell cycle, apoptosis, angiogenesis, signal transduction, inflammation, immunologic, and metabolic mechanisms. The molecular basis of antineoplastic roles of ABS depends on its proteomics, metabolomics, and transcriptomics features. ABS has antineoplastic effects on solid tumors like colon, bladder, breast, and osteosarcoma cancer cells. Also, ABS effects renal tubular apoptosis and has antitumoral roles on malign melanoma cells. ABS inhibits hematological tumors like myeloma and lymphoid cells. ABS induces apoptosis in retinal cells and has inhibitory effects on mesenchymal stem cells. It has an antiproliferative role on gastrointestinal tumors like hepatocellular carcinoma cells. Moreover, ABS has a treatment supportive role in cancer since it can prevent oxidative DNA damage and decrease the intestinal damage in necrotizing enterocolitis. Furthermore, it has chemopreventive and hepatoprotective features and can be used for prophylaxis and treatment of oral mucositis.

**Conclusion:**

ABS alters cell metabolism and cell cycle. ABS has antineoplastic role on cancer cells. The expanding context of ABS compromises anti-infective, antineoplastic, and wound healing features. ABS may also be used for the palliative, adjuvant, neoadjuvant, or supportive use by interventional radiology procedures for the treatment of solid tumors. Future controlled studies are necessary to clarify the pleiotropic role of ABS like antineoplastic, antithrombotic, anti-inflammatory, anti-infective, antifungal, and antioxidative effects.

## 1. Introduction

Ankaferd hemostat (ABS; Ankaferd Blood Stopper®) contains standardized plant extracts comprising Alpinia officinarum, Glycyrrhiza glabra, Thymus vulgaris, Urtica dioica, and Vitis vinifera [1]. These plant extracts have unique roles on the endothelium, blood cells, angiogenesis, cell growth, and cell mediators [2–4]. ABS especially was recognized for its hemostatic effect. ABS induces the creation of a protein network that has relationship between ABS and blood proteins, particularly with fibrinogen-gamma. Protein agglutination and erythroid aggregation are the two main mechanisms of ABS stimulated protein network. Spectrin, ankyrin, and actin are unique proteins which are controlled by ABS throughout erythroid aggregation course [5]. On the other hand, antineoplastic role of ABS was identified during the last decade. The aim of this paper is to review the molecular basis and associated clinical implications of the ABS as a topical antineoplastic agent.

## 2. Materials and Methods

Up to June 2022, literature searches were performed using the internet search engines Medline, Google Scholar, and Embase: Ankaferd. Only articles written in English were taken in the search. All abstracts were scanned. The studies that were found to be methodologically weak and not related with antineoplastic effects of Ankaferd were excluded. Articles in full text were assessed for eligibility and quality.Then, the qualitative synthesis included the following studies (Figure 1).

## 3. Molecular Basis of Antineoplastic Roles of Ankaferd Hemostat: Proteomics, Metabolomics, and Transcriptomics

ABS increases the level of various types of proteins and factors acting on cellular effects such as protein-2 (AP2), androgen receptor (AR), cyclic AMP response element or stimulating transcription factor-1 (CREATF1), cyclic AMP response element binding protein (CREB), E2F1–5, E2F6, EGR, interferon- (IFN-) stimulated response element (ISRE), Myc-Max, nuclear factor-1 (NF-1), protein53 (p53), SMAD2/3, peroxisome proliferator-activated receptor (PPAR), and Yin-Yang (YY1). These factors have important effects in several cellular processes, like control of the cell cycle, apoptosis, angiogenesis, signal transduction, inflammation, immunologic, and metabolic mechanisms [2].

Apoptosis seems to be the primary mechanism of action underlying antineoplastic effects of ABS. ABS can stimulate apoptosis in leukemia cells. Endothelial cell protein C receptor (EPCR) belongs to the activated protein C anticoagulant pathway. EPCR effect has not been completely clarified in various cell types where EPCR is known to be present, for example, hematopoietic cells and cerebral smooth muscle cells [6]. Protease-activated receptor 1 (PAR1) belongs to proteinase-activated receptor (PARs) family that present in seven transmembrane G-protein-coupled receptors group [7]. Stimulated PAR1 controls intracellular signaling by coupling G proteins. ABS modifies PAR1 and EPCR expression in K-562 and Jurkat cells in a time- and dose-dependent way. The role of PAR1 and p21 in this apoptotic mechanism was detected in Jurkat cells. ABS results in apoptosis via controlling PAR1- and p53-independent p21 involvement in apoptosis stimulation in leukemia cells, related with the concentration and duration of the application [8]. PAR1 has critical roles in hemostasis, inflammation, infection, apoptosis, and tumorigenesis. The effects of ABS on PAR-1 in the human umbilical vein endothelial cell (HUVEC) model and in relation to the “lipopolysaccharides- (LPS-) challenge” to endothelium were analyzed in a previous study [9]. In this study, ABS 10 *μ*L and 100 *μ*L had been given to HUVEC within the time periods of 5 minutes (min), 25 min, 50 min, 6 hours (h), and 24 h. The authors found dose-related reversible PAR1 decrease controlled via ABS inside the human umbilical vein endothelial cells. ABS-stimulated continuous PAR1 decreases with LPS. ABS is suggested as a topical biological response controller by altering PAR1 at the vascular endothelial and cellular level [9].

ABS has effects on colon cancer cells. The mechanism of antineoplastic effect of ABS over the Caco-2 colon cancer cells has been evaluated (Figures 2 and 3) [10]. ABS found to change glucose, fatty acids, and protein metabolisms. Also, ABS found to effect the cell cycle machinery. Besides, ABS stimulated critical cancer target and suppressor proteins such as carboxyl-terminal hydrolase 1, 60S ribosomal protein L5, Tumor protein D52-like2, karyopherin alpha 2, and protein deglycase DJ-1 were identified [10]. ABS has different effects on cancer targets and inhibitory proteins. ABS alters the cell metabolism and cell cycle in Caco-2 cells.

ABS has effects on renal tubular apoptosis. The effect of ABS, on renal tubular apoptosis and on expressions of endothelial nitric oxide synthase (eNOS), inducible nitric oxide synthase (iNOS), and apoptosis protease-activating factor-1 (Apaf-1) in the ipsilateral kidney was investigated [11]. ABS found to have a dual biphasic de novo effects on apoptosis. The challenge of severe hemorrhage in the renal tubular cellular microenvironment leads to ABS-stimulated decrease of the apoptotic molecules, suggesting that ABS can have role as a topical biological response controller.

ABS suggested to be a promising hemostatic agent in otology. Mucosal trauma stimulated apoptosis in guinea pig middle ear was investigated by comparing the hemostatic agents, absorbable gelatin sponge (AGS), microporous polysaccharide hemospheres (MPH), and ABS [12]. ABS and AGS groups showed lower epithelial thickness, inflammation, and capillary dilatation than did the control group. A reduction in Bcl-xl staining was detected in the middle ears of animals that were given MPH. Caspase 3 expression increased in the ABS and AGS groups than in the control group. Light microscopy clarified that ABS and AGS generate less inflammation and stimulated caspase expression that likely stimulate inflammatory cell apoptosis [12].

The resistance against chemotherapeutic drugs is a major problem in therapy of cancer. ABS has suggested to inhibit the development of melanoma cells, but mechanism is not yet fully clarified. ABS found to transfer some melanoma cell lines such as A2058 more sensitive to etoposide by changing the genes that have role in oxidative phosphorylation (OXPHOS) pathway [13]. ABS increases the sensitivity of A2058 against etoposide and has no effect against SK-MEL-5. The majority of the genes among oxidoreductase cluster found to take role in oxidative phosphorylation and electron transport chain [13]. The administration of ABS before etoposide may stimulate the response of melanoma cell lines because of the change of OXPHOS genes [13].

The antitumor effect of ABS on the MCF-7 breast cancer cell line was investigated [14]. The change of the levels of cancer-associated proteins of MCF-7 is upon application of ABS. Proteomic analysis clarified that ABS leads to an alteration in the levels of certain proteins including chaperones, p97, ATP5B, SELENBP1, PDIA6, and RPS10P5 [14]. ABS target certain proteins that were aberrantly expressed in breast cancer, especially the ER^+^ subtype [14].

ABS has effects on DNA, and it can prevent oxidative DNA damage [15]. In a previous study, the role of ABS on 8-hydroxy-2′-deoxyguanosine (8-OHdG), superoxide dismutase (SOD), and myeloperoxidase (MPO) levels over pleural adhesions in rabbits with pulmonary parenchymal damage was investigated [15]. The 8-OHdG levels were found to be lower in the ABS study group, and the differences between study and control groups were statistically significant (*p* < 0.001). The difference of SOD and MPO levels is not statistically significant between the groups [15]. The prevention of oxidative DNA damage by ABS was proven.

ABS effects apoptosis on retinal cells [16]. In a previous analysis, the cellular apoptotic roles of ABS on rabbit retina tissues were investigated. ABS was given into the vitreous of right eye of five rabbits. Oxidative injury, apoptosis, protein carbonylation, and DNA breakup were analyzed. In the ABS given eyes, sodium dodecyl sulphate polyacrylamide gel electrophoresis pattern of protein bands was stimulated; however, the other bands were decreased. Apoptosis was postponed, clarified by the morphological methods and caspase activity in the ABS administrated eyes. ABS stimulates protein carbonyle generation and DNA breakup were showed in the rabbit retina [16]. ABS showed to have an important role on apoptosis. ABS-related reductions of apoptosis in the retinal microenvironment showed that ABS may have a role as a topical biological response controller.

The antioxidant and antimutagenic features of ABS were investigated in a previous study [17]. The antioxidant effects were investigated using 2,2-diphenyl-1-picrylhydrazyl (DPPH) radical-scavenging and *β*-carotene-linoleic acid tests. The antimutagenic role was detected using the Ames Salmonella/microsome mutagenicity test with the bacterial mutant strains Salmonella typhimurium TA98 and TA100. ABS showed no free-radical-scavenging effects in DPPH assays at the analyzed concentrations; however, *β*-carotene-linoleic acid analysis revealed that ABS has total antioxidant activity rate of 47.06 ± 4.41%. Antimutagenic activity was found on TA100 at plate concentrations of 5%, 0.5%, and 0.05%, and on TA98 only at a plate concentration of 5%. ABS was proven to have antioxidant and antimutagenic features [17].

The proteomics, metabolomics, and transcriptomic of ABS are important to understand the molecular basis of antineoplastic effects of ABS. ABS has showed several pleiotropic roles, like antineoplastic and antimicrobial effects and tissue-healing features. Ankaferd's individual ingredients were clarified by the proteomic and chemical tests. ABS stimulates transcription of some transcription factors that is shown with transcriptomic analysis. ABS has showed cytotoxicity against human erythrocytes and tumoral cells in multiple myeloma, chronic myelogenous leukemia, and lymphoma [18–20]. Cyclic AMP response element-binding protein (CREB)/ATF BZIP transcription factor (CREBZF), PIAS-2, hepatocyte nuclear factor (HNF-4a), malic enzyme (ME-1), P18INK4C, and Midkine are the possible associated ingredients of ABS for this effect. ABS has shown to stimulate the expression of CREBZF resulting to the stimulation of the antineoplastic protein p53 [21]. HNF-4a has antineoplastic effects, and it is a component of ABS and might be partially responsible for its antitumorigenic effects [22]. ME-1 is an intracellular cytosolic protein, and it converts malic acid to pyruvic acid, creating nicotinamide adenine dinucleotide phosphate (NAPDH) [23, 24]. ME-1 has significant effects on cancer metabolism because NADPH is necessary for anaerobic respiration, and ME-1 level is found to be high in some cancers. ME-1 is also found in ABS. Midkine is a heparin-binding protein that has significant effect in tumoral angiogenesis, and its blockade can inhibit tumor growth [25, 26]. Protein inhibitor of activated signal transducer and activator of transcription- (PIAS-) 2 belong to the PIAS family, whose members inhibit the activity of the STAT proteins [27]. JAK-STAT signaling is an important pathway which has role in human carcinogenesis [28]. Cyclin-dependent kinase (CDK) inhibitor P18INK4C decreases tumorigenesis [29]. Its deficiency may cause tumor growth [30, 31]. CDKs are serine/threonine kinases which control the cell cycle. P18INK4C may have a role in the tumor-suppressor activity of ABS by suppressing CDKs. ABS has effects on the targets on cancer therapy like SND1, KPNA2, and PARK7. ABS upregulates the tumor suppressor proteins UCHL1 and RPL5. RPL5 stimulates the p53 apoptotic mechanism and leads to apoptosis [32].

ABS has several roles on transcriptomic also. ABS stimulates the transcription factors of AP2, AR, CREATF1, CREB, E2F1-5, E2F6, EGR, GATA, HNF1, ISRE, Myc-Max, NF1, NF-*κ*B, p53, PPAR, SMAD2/3, SP1, TRE/AP1, and YY1. These transcription factors control several biological mechanisms, like hemostasis, infection, cellular growth, and inflammation [33]. GATA controls erythroid differentiation and increases the erythroid proteins like spectin. GATA is found to be increased after ABS administration [33]. ABS increases the following transcription factors; AP2, AR, CRE-ATF1, CREB, E2F1-5, E2F6, EGR, ISRE, Myc-Max, NF1, NF-*κ*B, p53, PPAR, SMAD2/3, SP1, TRE/AP1, and YY1. These molecules have role in several stages of cellular growth, like control of cell cycle, signal transduction, angiogenesis, apoptosis, inflammation, acute phase reaction, immunity, and various metabolic molecular mechanisms [33].

## 4. Ankaferd Hemostat in Hematological Tumors

ABS has antineoplastic and cellular differentiation effects on the lymphoid cells [18]. ABS interacts tumor associated transcription factors. Effects of ABS on lymphoid neoplastic cells investigated in a previous study. ABS-treated B-CLL cells (at doses 0.5, 1 and 2 *μ*g/mL) stopped inflating, and more than half of tumor cells were died compared to 0.1 and 0.25 *μ*g/mL doses. Moreover, transformation of B-CLL cells to the blastic aggressive lymphoid forms was inhibited by ABS. ABS has antineoplastic effects at higher doses (>0.5 *μ*g/mL), and it stimulates the cellular differentiation at lower doses (<0.5 *μ*g/mL).

The role of ABS against myeloma cells in vitro and plasmocytoma generation in Balb/c mice was analyzed in vitro. The antineoplastic effect of ABS to the myeloma cells was detected by the 3-(4,5-dimethylthiazol-2-yl)-2,5-diphenyltetrazolium bromide-dye reduction assay [19].

## 5. Ankaferd Hemostat in Malign Melanoma

There is an unmet need for novel therapeutic and/or complementary methods in malign melanoma because the 5-year survival duration of metastatic melanoma patients is under 25% [34]. Plant extracts can have antineoplastic effects and can work synergistically with the conventional chemotherapeutics [35]. Melanocytes secrete “melanin” pigment. Melanocytes may transform into melanoma if their DNA injures [36]. The treatment response of nonmelanoma skin cancers to medical treatment is higher than melanoma. Melanoma cases have been rising nowadays, and nearly 53,000 people die annually worldwide because of melanoma [37]. ABS has antitumor effect on the primary melanoma cells and cell lines. In a recent study, the effect of ABS on dissimilar melanoma cell lines and primary cells was analyzed [35]. SK-MEL-10 (CVCL_6020), SK-MEL-9 (CVCL_U934), A2058 (ATCC® CRL-11147™), and MeWo (ATCC HTB-65™) melanoma cell lines were used in the study. These cells were given various amounts of ABS to detect the role of various dosages. An important reduction in cell viability against the control groups was detected in the cells that were treated with ABS. Also, increasing the concentration of ABS and the incubation during had a negative effect on cell viability. As a result, the antineoplastic effect of ABS on various melanoma cells has been proven [35].

In another study, cytotoxic, genotoxic, apoptotic, and reactive oxygen generating (ROS) effects of ABS were analyzed in the melanoma and normal cell lines. The cells were exposed to various concentrations of ABS (0.125 to 2%) for twenty-four hours. ABS was found to stimulate DNA injury, apoptosis, and ROS levels in both melanoma and normal cells in a dose-related way [38]. Moreover, these activities were considerably greater in melanoma cells than in normal cells.

## 6. Ankaferd Hemostat in Solid Tumors

ABS has antineoplastic effects on solid tumors [39]. The antineoplastic effects of ABS on osteosarcoma cell line (SAOS-2) survival and growth were investigated previously (Figure 4) [40]. Saos-2 which is generally used in drug resistance analyses was cultured in RPMI media containing 10% FCS, 1% pen/strep, and 1% sodium pyruvate. Then, cells were moved into 12-well tissue plates, in which 2, 4, 6, 8, and 10 *μ*L/mL concentrations of ABS solution were given to the stimulate medium. A control group was prepared in a fresh growth medium without ABS. Increase of the Saos-2 cells was followed-up for the 17 days during which yellow and opaque-like aggregates were detected in cultures increasing with ABS. A dose-dependent decrease was detected in cell proliferation, and a significant decrease was found in the survival of Saos-2 cells. Aggregate formation augmented after higher doses of ABS, and dose-related decrease was found in cell invasion [2]. ABS given Saos-2 osteosarcoma cells were detected to lose adhesion in vitro. A dose-related blockade in cell growth and an important decrease were found in the survival of SAOS-2 cells with ABS.

ABS has anticancer role also in colon cancer [10]. Currently, alcohol, N-butyl-2-cyanoacrylate, and caustic materials are utilized as tumor embolizers. In colon cancer liver metastases and hepatocellular cancer cases, ABS may be utilized for the palliative, adjuvant, neoadjuvant, or supportive role via interventional radiology methods for the treatment of solid tumors [41]. In a different study, the antineoplastic role of ABS on the colon cancer cells was identified [42]. After the administration of ABS to the culture medium, the decrease of cellular reproduction and loss in the viabilities of the human colon CaCo-2 cells were detected. The cultures were cultivated independently in 12-well tissue-culture containers where ABS with 2, 4, 6, 8, and 10 *μ*L/mL amounts was given to the culture medium. Cultivated cells without ABS in culture medium were prepared as a control group. The increase of CaCo-2 cells was followed-up for 16 days. ABS administration to culture medium leads to an increase in yellow and cloudy aggregates, together with enlarged amount of ABS. As a result, the inhibition of cellular reproduction and loss in the viabilities of the human colon CaCo-2 cells were associated with ABS concentrations *in vitro* (Figure 5) [42]. Another study regarding the Caco-2 cell also focused on the antineoplastic effects of ABS. The LC/MS-based proteomics technique was performed to analyze the role of ABS at the protein level [43]. The results were assessed with gene ontology, protein interaction, and pathway analysis. As a result of the study, ABS was found to alter glucose, fatty acids, and protein metabolism. Also, ABS has role in the cell cycle machinery. Furthermore, ABS was found to stimulate critical cancer target and suppressor proteins such as carboxyl-terminal hydrolase 1, 60S ribosomal protein L5, Tumor protein D52-like2, karyopherin alpha 2, and protein deglycase DJ-1 [43]. The proteomics results show that ABS affects various cancer targets and suppressor proteins. ABS has role on the cell metabolism and cell cycle in Caco-2 cells and indicates that ABS may be used as an antineoplastic treatment agent.

In a previous analysis, the molecular role of ABS on colon cancer was investigated. In the study, comparative analyses were performed with transcriptomic, proteomic, and metabolomic techniques on cancerous cells and untreated cancer cells in which antineoplastic effect was detected. As a result of this study, ABS was found to affect the biochemical processes happening in the cell with definite pathways. The levels of proteins such as Vinculin, Ezrin and HMGB1, that have roles in the mechanism of cancer, are altered by ABS and quantities of metabolites such as glutathione [44]. ABS affects several biological mechanisms as well as antioxidant activity and particularly cancer cell defense mechanisms.

ABS has also antineoplastic effects on bladder cancer. A previous study was conducted to analyze the antineoplastic role of ABS on bladder carcinoma in ex vivo patient tumor samples [45]. According to the results in the study, viability of cells decrease and the death rates of cells increased in statistically significant manner in bladder cancer cell cultures with ABS. Moreover, one of the main symptom of bladder cancer is bleeding. Therefore, the intravesical use of ABS may be beneficial, that has both haemorrhagic and antineoplastic features, in the control of patients with haematuria or postoperative bleeding after transurethral bladder resection. In the study, minimum 0.5 cm parts of fresh frozen tumor samples from patients with bladder tumor from 2015 to 2017 were collected. Primary bladder cancer cultures were collected from the frozen tumor samples. Two various doses of ABS were given on tumor cell cultures. Viability tests of each cell cultures were conducted. Flow cytometry was performed for the testing of apoptosis and necroptosis. Decreased cancer cell viability ratio in each ABS group compared with their own controls was found. Necroptosis was detected in the great majority of ABS groups, and necroptosis and apoptosis were found in some cell cultures [45]. The cytotoxic effect of ABS on bladder cancer cells was shown in the study. ABS may have potential for intravesical treatment agent for bladder cancer.

The role of ABS on breast cancer is also investigated in another study. Reduced cancer cell viability ratio in each ABS group against with their own controls was detected in a study [46]. Necroptosis was found in majority of ABS groups, and necroptosis and apoptosis were observed in breast cell cultures. The cytotoxic effect of ABS on breast cancer cells was well-demonstrated [46].

Being easily multiplication in vitro and having clinical usage potential in many fields primarily like hematopoietic stem cell transplants, regenerative medicine, tissue engineering, and gene therapy, mesenchymal stem cells pull attention. In a previous study, the contribution of stromal oriented mesenchymal stem cells (MSC) to the bleed stopping and wound healing effects of ABS is investigated in in vitro environment [47]. MSCs had been described by flow cytometry according to their differentiation potentials and surface antigen properties. Those MSC obtained from healthy bone marrow transplant donors grown in the DMEM-LG media having 10% fetal calf serum and 1% pen/strep. In the first group, ABS solution in 2, 4, 6, 8, 10, 25, 50, and 100 *μ*L/mL concentrations was added to the MSC cell groups which were confluent and grown in 12 pit tissue culture dishes. As a control group, cells to which medicine was not added and growing media were used. In the second group, by adding ABS solution to DMEM-LG having no serum, its effect to cells growth was investigated. Cells were followed for a period of 14 days. When liquid and homogenous ABS is added to the MSC growing media, aggregate formation was observed. It was observed that granule formation in cells showing adhesion or cells not sticking to culture dishes and aggregation was increased depending upon the ratio of ABS added to culture media. Since the cells have separated from the medium and have adhered to each other, further development steps could not be observed. Consequently, it is determined that ABS, when used in these ratios, affects culture media negatively on in vitro proliferation of MSCs due to intense aggregation (Figure 6) [47]. The effects of ABS in vitro in lower concentrations and its in vivo effects over cancer stem cell and in vivo stem cell dynamic need to be clarified.

## 7. Ankaferd Hemostat in Gastrointestinal Tumors

ABS has antineoplastic activity in hepatocellular carcinoma. In a previous analysis, HEPG2 hepatocellular carcinoma cells were given 8 *μ*L/mL of ABS for 24 hours, and the alterations were analyzed on both proteomic and genomic manners [48]. ABS did not decrease cell viability subsequent to 24 hours of the therapy but, and ABS inhibited cell viability after 72 hours. On the other hand, at the 24 hours of therapy with ABS, genomic and oncoproteomic tests showed diversification. Protein processing networks in endoplasmic reticulum that control protein folding, relocation, and degradation were altered by ABS. Moreover, mitochondrial apoptotic pathway can be stimulated by the hnRNP F-p53 interaction with the elongation of the ABS exposure period. ABS did not lead to P-glycoprotein-dependent drug resistance differently from several other used chemotherapeutics; therefore, ABS may also be used as combination treatment [48].

## 8. Ankaferd Hemostat as a Supportive Treatment of Cancer

ABS has chemopreventive, antioxidant, and supportive effects [49]. The chemopreventive role of ABS in 7,12-dimethylbenz[a]anthracene- (DMBA-) induced oral epithelial dysplasia is investigated in a previous study [49]. The buccal pouches of animals exposed to DMBA alone showed severe dysplasia; however, only mild or no dysplasia was found in DMBA + ABS group. ABS was also given to animals, and the control group revealed no dysplasia or other oral lesions [49]. The chemopreventive effect of ABS against DMBA-induced oral epithelial dysplasia was proven.

ABS is also beneficial in prophylaxis and treatment of oral mucositis [50]. In a previous study, the role of ABS in the prophylaxis and therapy of oral mucositis in patients who were given chemotherapy in childhood was investigated. In the study, citrulline which is a biochemical marker for mucosal barrier damage was analyzed, and the role of ABS treatment in mucositis was related to quantitative data along with the clinical findings. There was no important difference between the chemotherapy courses given with standard oral care (SOC) and with ABS plus SOC before chemotherapy, but an important difference was found between these courses after chemotherapy about stages of oral mucositis. The extent of the reduction in serum citrulline levels was found to be higher in the chemotherapy courses with SOC than in those with SOC plus ABS. As a result, ABS was considered as an effective agent for the prophylaxis and therapy of oral mucositis secondary to chemotherapy in childhood cancers [50].

On the other hand, ABS is also effective in chemotherapy-induced oral mucositis in adult population [51]. Oral mucositis is one of the most severe complications of anticancer therapy that affects 40-80% of cancer patients. The safety and efficacy of ABS in the management of chemotherapy-related oral mucositis in patients with hematological malignancies are analyzed previously. ABS was administrated to the patients with grade 3-4 mucositis. After the patients' mouthwash and swallow the five milliliters of ABS, the healing time was calculated. Median healing time was found as 6.6 days [51]. As a result, ABS can play an important role in the therapy of chemotherapy-associated severe oral mucositis in patients with hematological malignancies.

In another study, the chemopreventive role of ABS in 7,12-dimethylbenz[a]anthracene (DMBA) is related oral epithelial dysplasia. The buccal pouches of animals given DMBA alone showed up dysplasia while only moderate or no dysplasia was found in DMBA + ABS group [49].

Necrotizing enterocolitis (NEC) is an important health problem that leads to morbidity and mortality. Risk factors for NEC include prematurity, oxidative stress, inflammation, and apoptosis. Whether treatment with ABS decreased the severity of NEC in rat pups in an experimental NEC model is investigated. Total oxidant status, oxidative stress index, tumor necrosis factor *α* and interleukin-1*β* levels, lipid, protein, and deoxyribonucleic acid oxidation products were lower in the NEC + ABS group compared to NEC + saline group while total antioxidant status, glutathione, and superoxide dismutase levels were higher in the NEC + ABS group. ABS found to decrease the intestinal damage in NEC due to its antioxidant, anti-inflammatory, and antiapoptotic features [52].

ABS also has hepatoprotective features [53, 54]. In previous studies on the trace element and vitamin content of ABS, Akar et al. analyzed the Fe (III), Cu (II), Zn (II), and Ag (I) ions in ABS. Concentrations were 2163 ± 7, 2.56, 9.2, and 45.0 ppm, respectively, which indicates an association between high iron levels and the hemostatic action of ABS [55]. The absence of Pb (II), Ni (II), Cr (IV), Co (II), and Cd (II) ions in ABS was also shown [55]. Koluman et al. found various antioxidant molecules in ABS, such as vitamin E [56]. Akişin and Akar found the zinc content of ABS and the association between high zinc levels and the wound healing action of ABS [57]. Because of the antioxidative and hepatoprotective roles of the trace elements and vitamins like magnesium, calcium, vitamin D, vitamin B12, vitamin B9, vitamin A, and vitamin E [58–61]; antioxidative, antiinflammatory, and hepatoprotective roles of ABS may be related with its trace elements and vitamins.

## 9. Future Perspectives on Ankaferd Hemostat as a Topical Biological Response Modifier

ABS has hemostatic roles in bleedings and has several pleiotropic effects. The quick generation of a protein network, most importantly fibrinogen gamma, with the erythrocyte aggregation is responsible for the hemostatic role of ABS. The whole mechanism involves ABS-stimulated generation of the protein network by vital erythrocyte aggregation. Vital erythrocyte aggregation happens with the help of spectrin, ankyrin, and actin proteins on the membrane of the erythrocytes. ABS most importantly alters cell metabolism and cell cycle. ABS has antineoplastic role on cancer cells. The expanding context of ABS compromises anti-infective, antineoplastic, and wound healing features. ABS is generally used for to provide hemostasis and stimulate wound healing. However, ABS may also be used for the palliative, adjuvant, neoadjuvant, or supportive use by interventional radiology procedures for the treatment of solid tumors. This theory may be analyzed in future clinical studies. Furthermore, future controlled studies are necessary to clarify the pleiotropic role of ABS like antineoplastic, antithrombotic, anti-inflammatory, anti-infective, antifungal, and antioxidative effects.

## Figures and Tables

**Figure 1:** The PRISMA flow diagram for the Ankaferd search.

**Figure 2:** The scheme of downregulated (a) and upregulated (b) proteins after Ankaferd hemostat (ABS) given on the human colon cancer cell line, CACO-2 (reproduced with the open access policy of the Journal; Bio Med Res (https://www.hindawi.com/journals/bmri/2019/5268031/fig 4/).

**Figure 3:** The classification of upregulated proteins in cellular component (a), in organelles (b), and in cellular processes (c) after Ankaferd hemostat (ABS) given on the human colon cancer cell line, CACO-2 (reproduced with the open access policy of the Journal; Bio Med Res (https://www.hindawi.com/journals/bmri/2019/5268031/fig 3/).

**Figure 4:** The inhibitory effect of Ankaferd Hemostat (ABS) on the Saos-2 cells. (a) The control group without ABS (10× magnification). (b) 10 *μ*L ABS given Saos-2 cells (10× magnification) at the seventeenth day.

**Figure 5:** The inhibitory effect of Ankaferd Hemostat (ABS) on the CaCo-2 cells. (a) The control group without ABS (10× magnification). (b) 10 *μ*L ABS given CaCo-2 cells (10× magnification) at the sixteenth day.

**Figure 6:** In vitro proliferation of the MSCs was negatively affected by Ankaferd Hemostat (ABS) due to intense aggregation. (a) The control group without ABS (10× magnification). (b) 10 *μ*L ABS given mesenchymal stem cells (10× magnification) at the fourteenth day.

## Data Availability

The data supporting this systematic review are from previously reported studies and datasets, which have been cited. The processed data are available from the corresponding author upon request.
